The article "Sustainable Trend of Big Data in Enterprise Supply Chain Under the Artificial Intelligence Green Financial System" was retracted in 2023. Reasons: unreliable results or conclusions; concerns about the data; concerns about the peer review; concerns about the citations.

# Sustainable Trend of Big Data in Enterprise Supply Chain Under the Artificial Intelligence Green Financial System

**DOI:** 10.1155/2022/3065435

**Published:** 2022-10-11

**Authors:** He Wu, Xuancheng Zhang, Yiqin Wang

**Affiliations:** ^1^School of Economics, Jilin University, Changchun 130000, Jilin, China; ^2^Northeast Asian Studies College, Jilin University, Changchun 130000, Jilin, China; ^3^School of Marxism, Jilin Business University, Changchun 130000, Jilin, China

## Abstract

Today, with the rapid development of the Internet, society has entered the era of “information explosion.” Financial data are a particularly important part of network information, and it has also reached a new level of public demand. The frequent appearance of words such as “carbon peak” and “green” indicates the transition of national policies to the field of sustainable development. Sustainable development would become an inevitable choice, and a green supply chain has become a new trend under this policy background. Supply chain finance uses the ideas and methods of key supply management to provide financial services to related enterprises. If an enterprise cannot acquire, organize, and use the information and data in the supply chain, it is likely to be outdated or even abandoned in the short term. This paper takes the artificial intelligence green financial system as the background and uses the cooperation theory model to analyze and predict the big data information of the enterprise supply chain. It realizes the transformation of information into sustainable resources for enterprises and releases the huge potential of big data. In this model, this model not only helped the company's overall profit increase by about 8.79% but also provided scientific support for corporate decision-making and promoted the development of the company.

## 1. Introduction

At present, “green supply chain finance” has become a hot topic. It can be seen that the three words green, sustainable, and double carbon contained in the current supply chain finance industry indicate that these words have firmly grasped the “core” of the current supply chain finance development. Supply chain finance provides financial services for the real economy and is gradually moving from silent accumulation to the front. This requirement is even more urgent, particularly during the crucial time when supply-side structural change and the transformation of both new and old kinetic energy are being promoted.

There is scholars' related research on supply chain finance now: Kouvelis proposed that supply chain finance was a model in which two or more organizations in the supply chain finance composed of external service providers plan, execute, and control the flow of financial resources between organizations so as to achieve the purpose of jointly creating value [1]. Martin and Hofmann believed that supply chain finance literally mean the integration and innovation of supply chain and finance [2]. Thomas believed that supply chain finance was a financing activity, and the leading enterprises on the chain were crucial and played a huge role in capital transactions. Financing activities traditionally used fixed assets as mortgages. Under supply chain finance, enterprises mortgage current assets such as accounts payable, prepayments, and inventories to financial institutions, which have nothing to do with fixed assets [3]. Song et al. found that supply chain finance came into being, mainly because it combined the real economy with financial issues to meet the capital needs of SMEs. It reduced the risk of financial institutions, saved business development costs, improved the efficiency of institutional operations, and drove the development of the market economy to a greater extent [4]. Chen and Xu believed that supply chain finance was the use of financing, risk reduction, and other means and technologies to optimize the management of working capital in the supply chain process and transaction process and to effectively use liquid investment funds [5]. Yan proposed that supply chain finance relied on the core enterprise credit with advantages in the industrial chain and effectively integrated the information flow, logistics, and capital flow between enterprises in the supply chain so as to provide financial services for the upstream and downstream procurement and production and sales process of core enterprises [6]. Simply put, supply chain finance refers to the practice of banks using the products and services offered by their main businesses as well as upstream and downstream companies as solvents to boost their liquidity.

The article "Sustainable Trend of Big Data in Enterprise Supply Chain Under the Artificial Intelligence Green Financial System" was retracted in 2023. Reasons: unreliable results or conclusions; concerns about the data; concerns about the peer review; concerns about the citations.

There are scholars related to artificial intelligence research now: Hassabis et al. proposed that an expanding field of technology called artificial intelligence researched and developed a variety of ideas, approaches, tools, and software programs that imitated, enhanced, and extended human intellect [7]. Miller found through research that artificial intelligence was rising in the field of computing and has been widely used in various aspects, such as robot technology, economy, political decision-making, control system, simulation system, and other fields [8]. Institute M believed that artificial intelligence was a discipline that studies how to make computers do intelligent work that could only be performed by humans before. The underlying tenet and core ideas of the field of artificial intelligence were reflected in this phrase [9]. Krittanawong et al. believed that building artificial systems with specific intelligence and studying the rules governing human intellect were both considered to be forms of artificial intelligence. It looked at ways to program computers to perform tasks calling for the human intellect. That was how to use computer hardware and software to imitate certain fundamental ideas, practices, and strategies of intelligent human behavior [10]. Rongpeng believed that the goal of artificial intelligence, a subfield of computer science, was to comprehend intelligence and develop new kinds of intelligent robots that can react similarly to human intelligence [11]. Various research found that since the 1970s, artificial intelligence has been regarded as one of the three leading technologies of space technology, energy technology, and artificial intelligence, and it was also regarded as the three core technologies of genetic engineering, nanoscience, and artificial intelligence in the 21^st^ century [12]. Generally speaking, making robots capable of doing complicated tasks that typically needed human intelligence was one of the primary research objectives of artificial intelligence. However, various individuals and periods have different perspectives on this “difficult labor.”

In today's increasingly developed Internet, the market competition of core enterprises is becoming increasingly fierce, therefore the primary objective of today's key businesses was to have an efficient and dependable supply chain [13]. The integration of the Internet, artificial intelligence, and supply chain finance has brought about a favorable impact on the sustainable development enterprises. With the help of the Internet platform to achieve information integration, the Internet collected information and data for sharing greatly improves the financial operation efficiency of the supply chain, while ensuring capital security. Supply chain finance came into being and gradually penetrated various fields that enterprises needed to innovate and develop. It helped to improve the competitiveness of enterprises, and then new financing channels for small and medium-sized enterprises emerged as the times require. At present, the scope of application of supply chain finance is gradually expanding, supply chain finance is gradually entering a period of renewal, and the emergence of Internet technology has provided a new development opportunity for supply chain finance.

## 2. Big Data Application in Supply Chain

### 2.1. Overall Characteristics of the Big Data in Supply Chain

#### 2.1.1. Supply Chain Strategic Decision

Big data analysis provides precise information about an organization for enterprises to make strategic decisions [14]. Big data, for example, can provide precise information on any return on investment and provide insight into potential suppliers. The strategic procurement decision should take into account not only various procurement factors but also the strategic capabilities of suppliers [15]. Big data processing capability is an evaluation factor in the selection of supply chain partners. To weed out supply chain partners that can adapt to future big data difficulties, the analytical hierarchy process (AHP) and fuzzy comprehensive assessment approaches are applied [16]. Big data analysis has recently attracted a lot of interest in the field of product creation. Big data analysis can increase product flexibility and product designers' self-assurance. Customers' purchase history and online behavior are obtained from customers big data. In important industries, the value of big data manifests in the use of customer opinion data polarity to identify product characteristics and predict trends. The significant role of big data analysis summarized in this paper is shown in Figure 1.

The article "Sustainable Trend of Big Data in Enterprise Supply Chain Under the Artificial Intelligence Green Financial System" was retracted in 2023. Reasons: unreliable results or conclusions; concerns about the data; concerns about the peer review; concerns about the citations.

#### 2.1.2. Supply Chain Network Design

Big data analysis of supply chain network design enable enterprises to gain an advantage in the competition. Large randomly generated datasets in mixed-integer nonlinear models are exploited to screen distribution center locations and assume that intelligent marketing intelligence tools are leveraged to analyze behavioral datasets [17]. The findings have demonstrated that big data analysis may collect extra client information, opening up prospects for sophisticated distribution network design [18].

#### 2.1.3. Supply Chain Agility and Sustainability

At present, numerous scholars have conducted research on the agility of advanced supply chains and the sustainability of supply chains. Using as an illustration of the multi-objective mathematical model of green supply chain management, it not only integrates big data science to collect data and control data quality but also integrates social media data and company financial and operational data to effectively combine them [19]. Additionally, using expert judgment can help industrial growth be more resilient to risks and uncertainties and improve long-term sustainability.

### 2.2. Big Data Throughout the Supply Chain Process

Following a search of the database's pertinent literature, it is discovered that the supply chain industry's big data analysis focuses on strategic decision-making, network design, agility, and sustainability [20]. The big data analysis of the supply chain process mainly focuses on demand planning, procurement and production, inventory, and logistics distribution, etc. [21], as shown in Figure 2.

The article "Sustainable Trend of Big Data in Enterprise Supply Chain Under the Artificial Intelligence Green Financial System" was retracted in 2023. Reasons: unreliable results or conclusions; concerns about the data; concerns about the peer review; concerns about the citations.

### 2.3. Big Data Applications in Supply Chains of Different Industries

Currently, one of the common goals, when big data are applied to supply chains of many sectors, is to make excellent use of data and increase productivity by giving accurate information to accurate users in a timely way [22]. Big data analysis have been used in different industrial supply chains, including finance, technology, medical care, consumption, energy, and manufacturing. Each of them has a unique data processing and commercial value, as shown in Figure 3:

According to the big data analysis survey and statistics in Figure 3, the proportion of the supply chain in the banking and financial industries is nearly half, which shows that they attach great importance to the application of big data. The supply chain of the high-tech industry has a relatively high proportion, ranking second and accounting for about 14%. The second proportion from high to low is medical care, consumption, energy, manufacturing supply chain, etc.

In view of the statistical data shown in Figure 3, this paper obtains the commercial value of big data for different industries by further reading related literature.

Table 1 shows the application status and commercial value of big data in industrial supply chains such as banking, technology, medical care, consumption, energy, and manufacturing. For example, data processing in manufacturing/high-tech industries for product failure analysis, patent record retrieval, and intelligent location provide business value for product optimization, cost reduction, and rapid problem resolution. It is precise because of this that big data can show its value in this industry.

The above analysis results show that various industries around the world regard the realization of big data analysis applications as an extremely important development direction, especially for data-oriented industries, the realization of its applications has become very necessary.

## 3. Big Data Benefit Model of Green Supply Chain Finance

Establishing a big data benefit model of green supply chain finance and using the replication dynamic equation method to study the impact of big data sustainability, provides an effective way to promote small and medium-sized enterprises in the upstream supply chain to use environmental management strategies to carry out production [23]. In this paper, the green degree improvement *X* of the entire supply chain is taken as the research variable. This paper builds a financial big data benefit model of a green supply chain to study the decision-making problem of member enterprises in any supply chain under the condition of specific financial budget constraints. The aspects of demand planning, purchasing, production, inventory, and logistics and distribution are represented by variable y_*i*_. The constructed model is as follows:

(1) $$\begin{array}{c} S_{i}\left(X,y_{i}\right)=A-\beta X^{-\gamma }y_{i}^{-\delta }\text{.} \end{array}$$

Among them, the supply chain member companies are represented by *S*_*i*_, and the sales effort invested by the company is represented by y_*i*_. The greenness level of the entire supply chain is represented by *X*, and the greenness improvement contributed by the enterprise supply chain is represented by *x*_*i*_. The maximum market capacity of enterprise supply chain products is represented by A, and *π*_i_ is the income of the enterprise. The following studies the decision variables *X* and y_*i*_ of each firm *i* when it reaches equilibrium and solves the following constraint maximization problem:

(2) $$\begin{array}{c} \max_{X\;y_{i}}\pi_{i}=m_{i}\left(A-\beta X^{-\gamma }y_{i}^{-\delta }\right)\\ s.t.\varphi \left(x_{i}{,y}_{i}\right):hx_{i}+ky_{i}=B_{i}\text{.} \end{array}$$

Among them, *h* > 0, *k* > 0, *B*_*i*_ > 0.*i*=1,2, ⋯, *n*. The Lagrangian function constructed according to the above formula is as follows:

(3) $$\begin{array}{c} L\left(X,y_{i}\right)=m_{i}\left(A-\beta X^{-\gamma }y_{i}^{-\delta }\right)-\mu \left(hx_{i}+ky_{i}-B_{i}\right)\text{.} \end{array}$$

The first-order condition is solved. Among them, *x*_*i*_=*X* − ∑*x*_−*i*_, so *∂L*/*∂X*=*∂L*/*∂x*_*i*_, and the gradient vector ∇*φ*(*X*^*∗*^, *y*_*i*_)=(*h*, *k*) of the constraint is not 0, so there are

(4) $$\begin{array}{c} m_{i}\beta \gamma y_{i}^{-\delta }X^{-\gamma -1}-\mu h=0\text{,}\\ m_{i}\beta \delta y_{i}^{-\delta -1}X^{-\gamma }-\mu k=0 \end{array}$$

It can be got that

(5) $$\begin{array}{c} X^{*}=\frac{\gamma k}{\delta h}y_{i}\text{,}\\ y^{*}=\frac{1}{k}\left(B_{i}-hx_{i_{i}}^{*}\right) \end{array}$$

The reaction function between the enterprise *i* and other members is obtained by eliminating constraint *y*_*i*_

(6) $$\begin{array}{c} X^{*}=\frac{\gamma B_{i}}{h\left(\delta +\gamma \right)}-\frac{\delta }{\delta +\gamma }\sum x_{{-}_{i}}\text{.} \end{array}$$

Taking Formula (6) for the partial derivative function respectively, it can be got

(7) $$\begin{array}{c} \frac{\partial x_{i_{i}}^{*}}{\partial h}=-\frac{\gamma B_{i}}{\left(\delta +\gamma \right)h^{2}}<0\text{,}\\ \frac{\partial x_{i_{i}}^{*}}{\partial \gamma }=-\frac{\delta }{{\left(\delta +\gamma \right)}^{2}}\left[\frac{B_{i}}{h}+\sum x_{-i}\right]>0\text{,}\\ \frac{\partial x_{i_{i}}^{*}}{\partial \delta }=-\frac{\gamma }{{\left(\delta +\gamma \right)}^{2}}\left[\frac{B_{i}}{h}+\sum x_{-i}\right]<0\text{.} \end{array}$$

The objective function of this supply chain should be expressed as follows:

(8) $$\begin{array}{c} \max_{X\;,y_{i}}\overset{n}{\underset{i=1}{\sum }}\pi_{i}=\overset{n}{\underset{i=1}{\sum }}m_{i}\left(A-\beta X^{-\gamma }y_{i}^{-\delta }\right),i=1,2,\cdots ,n\text{,}\\ s.t.g\left(X,y_{1},\cdots ,y_{n}\right):hX+k\overset{n}{\underset{i=1}{\sum }}y{}_{i}=\overset{n}{\underset{i=1}{\sum }}B_{i}\text{.} \end{array}$$

In order to solve the optimization problem defined by the above equation, a Lagrangian function is constructed, namely

(9) $$\begin{array}{c} \tilde{L}\left(X,y_{i}\right)=\overset{n}{\underset{i=1}{\sum }}m_{i}\left(A-\beta X^{-\gamma }y_{i}^{-\delta }\right)-\mu_{1}\left(hX+k\sum y_{i}-\sum B_{i}\right)\text{.} \end{array}$$

The first-order condition is solved by $\partial \tilde{L}/\partial X=0,\partial \tilde{L}/\partial y_{i}=0,i=1,2,\cdots ,n$. Taking the product form of the matrix to simplify the expression, it is expressed as follows:

(10) $$\begin{array}{c} \beta \gamma X^{-\gamma -1}.\overset{n}{\underset{i=1}{\sum }}m_{i}y_{i}^{-\delta }-\mu_{1}h=0\text{,}\\ \beta \delta X^{-\gamma }•\left[\begin{array}{c} m_{1}y_{1}^{-\delta -1}\\ \vdots \\ m_{n}y_{n}^{-\delta -1} \end{array}\right]=\left[\begin{array}{c} \mu_{1}k\\ \vdots \\ \mu_{n}k \end{array}\right]\text{.} \end{array}$$

Combined with the elimination of constraints, the following equations can be obtained:

(11) $$\begin{array}{c} X^{**}=\frac{\gamma k}{\delta h}\sum y_{i}=\frac{\gamma }{h\left(\delta +\gamma \right)}\sum B_{i}\text{,}\\ X_{*I*}^{**}=\frac{\gamma }{h\left(\delta +\gamma \right)}\sum B_{i}-\sum x_{-i}\text{.} \end{array}$$

Let *t*=∑*B*_*i*_/*B*_*i*_, *α*=*X*^*∗*^/*x*_*i*_^*∗*^, when *t* > *α*, after the entire supply chain achieves Pareto equilibrium, the total green degree *X*^*∗∗*^ is greater than the total green degree improvement *X*^*∗∗*^ when any of its enterprises reach equilibrium.

The article "Sustainable Trend of Big Data in Enterprise Supply Chain Under the Artificial Intelligence Green Financial System" was retracted in 2023. Reasons: unreliable results or conclusions; concerns about the data; concerns about the peer review; concerns about the citations.

It can be obtained by calculation as follows:

(12) $$\begin{array}{c} \frac{X^{**}}{X^{*}}=\frac{t\left(\alpha \delta +\gamma \right)}{\alpha \left(\delta +\gamma \right)}\text{.} \end{array}$$

## 4. Evolutionary Model Stability

The high cost of third-party financing resources would increase the cost burden of upstream SMEs in the supply chain. So, for SMEs in the upstream supply chain, using green supply chain finance services has become the best course of action. From the model results, SMEs can choose to take green financial measures or not. Correspondingly, for upstream SMEs of different levels, core companies also adopt two strategic results when applying for supply chain financing, one is to provide guarantees to upstream SMEs, and the other is to have no guarantees. The final result of the strategic combination of core enterprises and SMEs is shown in Table 2.

Among them, assuming that *y* represents the probability that upstream small enterprises choose “take”. *x* represents the probability that core enterprises choose “guarantee.” Figure 4 shows the dynamic trend and equilibrium of the core enterprise group under the three conditions of *y*=*y*_0_, *y* > *y*_0_, and *y* < *y*_0_. When *y*=*y*_0_, then *F*(0)=0, and *x* is in a stable state at this time. That is, when the possibility of SMEs “taking” response is 0, there is no difference in the choice of “guarantee” and “no guarantee” for core enterprises. That is, when the possibility of SMEs' “taking” response is zero, the core enterprises have no difference in the “guarantee” and “no guarantee” response options.

If *x*=*x*_0_, then *F*(0)=0, then *y* is in a stable state. That is, when the “guarantee” response possibility of the core enterprise is 0, there is no difference between the “take” and “not take” response choices of SMEs, as shown in Figure 5.

In the same coordinate system, the dynamic phase diagram of the core enterprises and their upstream SMEs is drawn, as shown in Figure 6.

By examining the dynamic evolution process of the asymmetric replication process between core enterprises and their upstream SMEs, the following four equilibria are obtained:

When the result is in the area ①, *x* > *x*_0_ and *y* > *y*_0_, then the deductive equilibrium point *x*=0, *y*=1 is that the core enterprise and its upstream SMEs would definitely choose the strategy combination of not to guarantee or adopt.

When the result is in the area ②, *x* < *x*_0_ and *y* < *y*_0_, then the deductive equilibrium point *x*=0, *y*=0 is that the core enterprise and its upstream SMEs would definitely choose the strategy combination of not to guarantee or not to adopt.

When the result is in the area ③, *x* < *x*_0_ and *y* > *y*_0_, then the deductive equilibrium point *x*=1, *y*=0 is that the core enterprise and its upstream SMEs would definitely choose the strategy combination of guaranteeing or not to adopt.

When the result is in the area ④, *x* > *x*_0_ and *y* > *y*_0_, then the deductive equilibrium point *x*=1, *y*=1 is that the core enterprise and its upstream SMEs would definitely choose the strategy combination of guaranteeing or adopting.

It is concluded from this that through the sustainable trend analysis of big data in the enterprise supply chain under the artificial intelligence green financial system, the enterprise strategy adopted under this model can increase the overall profit of the enterprise by 8.79%. In order to promote enterprises to implement green supply chain finance in the artificial intelligence green financial system, it is necessary for core enterprises to optimize their guarantee strategies. On the one hand, it is necessary to increase the proportion of guarantees provided for upstream SMEs when they implement management strategies for production and reduce the proportion of upstream SMEs that do not implement management strategies to implement management. The development of green supply chains and the promotion of green supply chain finance should be the primary concerns of core businesses. The core enterprises should concentrate on promoting the development of green supply chain finance and green supply chain so that the stakeholders of green supply chain finance can see the long-term benefits of green supply chain finance at the same time, not just the immediate short-term benefits. This would allow the relevant stakeholders of green supply chain finance to see another aspect. Let stakeholders of green supply chain finance not only see the long-term benefits of green supply chain finance but also the short-term benefits.

The article "Sustainable Trend of Big Data in Enterprise Supply Chain Under the Artificial Intelligence Green Financial System" was retracted in 2023. Reasons: unreliable results or conclusions; concerns about the data; concerns about the peer review; concerns about the citations.

## 5. Suggestions for Green Supply Chain Big Data

### 5.1. Green Supply Chain Finance Supports the Growth of the Green Supply Chain

To effectively promote green supply chain management, it is important to thoroughly comprehend the function that green supply chain finance plays. It is also required to update pertinent laws and policies regarding green supply chain finance and increase the impact of this sector. The promotion of green supply chain management is still plagued by two major issues. First, small and medium-sized manufacturers upstream in the supply chain are hesitant to incorporate environmental protection into the production process because they want to maximize profits and have limited resources. Second, manufacturers who implement ecological supply chain management are faced with the dilemma of a shortage of funds because they invest part of their funds in environmental protection work. The implementation of an ecological supply chain finance strategy can not only promote upstream SMEs to use environmental management strategies to carry out production but also provide new financing channels for enterprises that use ecological supply chain management strategies, thereby promoting ecological supply chain management from the capital level. It further promotes the green supply chain management from the financial level. In this regard, the government should also improve the laws, regulations, and policies related to ecological supply chain finance and promote the implementation and development of the ecological supply chain finance strategy through policy guidance to enhance its influence.

The article "Sustainable Trend of Big Data in Enterprise Supply Chain Under the Artificial Intelligence Green Financial System" was retracted in 2023. Reasons: unreliable results or conclusions; concerns about the data; concerns about the peer review; concerns about the citations.

### 5.2. Enhancing the Participation of Green Supply Chain Financiers

The main stakeholders of ecological supply chain finance are commercial banks, core enterprises, and small and medium-sized enterprises upstream of the supply chain. In addition, most core enterprises pay less attention to environmental pollution when financing. By establishing an evolutionary game model between core enterprises and their upstream SMEs and a noncooperative game model between commercial banks and core enterprises to verify the strategy that commercial banks, core enterprises, and upstream SMEs jointly participate in green supply chain financing so as to increase the enthusiasm of key stakeholders to participate.

### 5.3. Intelligent Risk Control Using Big Data to Achieve Risk Prevention and Control in Key Links

For the intensive legal compliance audit points, the procurement process and the implementation of material audit only rely on manual auditing and selection by procurement personnel, which results in a large workload. It is not conducive in improving the efficiency and quality of procurement and even leads to the risk of a clean government, which does not meet the current legal and compliant construction needs. Therefore, it is urgent to introduce big data processing capabilities to replace manpower to carry out procurement risk prevention and control. Big data are applied to risk prevention and control mechanisms such as pre-event control, in-event supervision, and post-event analysis to achieve safety compliance.

Data fields such as product name, material name, supplier name, and item name should be obtained through monitoring, as well as the property amount limits control mode, total quota, execution quota, budget quota, payment type, order number, material code, commodity price, and contract number code when performing the contract. Other data fields, such as product catalog decision-making information should be used to enforce the control of violations and refuse to execute violations.

### 5.4. Intelligent Prediction to Realize Automatic Identification of Unstructured Data Risks

The traditional procurement model is “demand-oriented,” and there are management difficulties such as slow demand response and imprecise demand planning. Relying on big data analysis capabilities to change the way of demand response is the way demand-driven supply has been transformed into an active stocking to break the bottleneck of various professional systems and make data transparent and visualized. The correlation of demand, purchasing, supply, and sales forecasts is realized through data analysis and combined with the current inventory and purchasing cycle to realize active stocking. It significantly improves demand planning and procurement planning accuracy, further enhancing supply chain agility and demand responsiveness. Taking materials as an example, the key data in the supply chain system and the important data in the branch system are integrated, monitored, and analyzed by big data so as to grasp the market trend and identify bottlenecks and deal with them in time. Through big data analysis, the sales department can guide orders and stock up reasonably so as to avoid untimely supply or stagnant inventory that deviates from monitoring and sales. They can guide the network department to adjust the installation and maintenance capabilities and effectively guarantee business development.

The article "Sustainable Trend of Big Data in Enterprise Supply Chain Under the Artificial Intelligence Green Financial System" was retracted in 2023. Reasons: unreliable results or conclusions; concerns about the data; concerns about the peer review; concerns about the citations.

Texts such as procurement documents and bids/receipts are standardized, and they are used to explore the value of parseable unstructured data. Then big data automated sharing tools are used to certify supplier qualifications for bid attachments. Monitoring the abnormal situation of expert scores can ensure that enterprises can legally implement various procurements and reduce and avoid legal and integrity risks.

### 5.5. Intelligent Operation to Promote the Improvement of Supply Chain Efficiency

Most of the traditional statistical analysis methods for indicators are to obtain the raw data of each system. The data are processed through EXCEL, and the statistical results of the indicators are counted. Its calculation process is complicated, and due to the statistical cycle, the data have a lag, which cannot meet the needs of real-time control and tracking of index results. By building a big data analysis system, data can be deeply excavated and presented in real time, such as comprehensive statistical analysis of key procurement indicator data so as to have an accurate and timely grasp of the business development in the supply chain. It can also conduct in-depth and specific analysis to find out key influencing indicators and provide data support for subsequent judgment and decision-making.

## 6. Conclusion

On the basis of replicating dynamic equations, this paper used the static game method of complete information to construct cooperative and noncooperative evolutionary game models of core enterprises and small and medium-sized enterprises. In order to better promote the development of green supply chain finance, it is combined with financing methods. By analyzing the individual interests and overall interests of core enterprises and small and medium-sized enterprises in cooperation and noncooperation, this paper has proved that it is very necessary for core enterprises and small and medium-sized enterprises to carry out green supply chain finance. It also provided directions for the further development of green supply chain finance and the promotion of green supply chain data management, and at the same time providing constructive suggestions for sustainable development strategies in the implementation and development of green supply chain finance.

The article "Sustainable Trend of Big Data in Enterprise Supply Chain Under the Artificial Intelligence Green Financial System" was retracted in 2023. Reasons: unreliable results or conclusions; concerns about the data; concerns about the peer review; concerns about the citations.

## Figures and Tables

**Figure 1:** Role of big data analysis.

**Figure 2:** Applications of big data analysis in the supply chain.

**Figure 3:** Application of big data analysis in the supply chain of different industries.

**Figure 4:** Replication dynamic phase diagram of the core enterprise group.

**Figure 5:** Phase diagram of replication dynamics of SME groups.

**Figure 6:** Evolutionary trajectory map between core enterprises and their upstream SMEs in the supply chain.

**Table 1:** Application of big data in the supply chain of banking, science and technology, medical care, consumption, energy, and manufacturing industries.

	Data processing mode	Commercial value
Banking/Finance	Market evaluation new product risk assessment	Increase market value, improve customer loyalty, increase overall revenue, and reduce financial risk
High-tech	Comprehensive product analysis, patent record retrieval, smart device global positioning location service	Optimize products, design and manufacture to reduce warranty costs, and speed up problem-solving
Medical care	Shared medical records, accelerated diagnosis, and telemedicine	Improved diagnostic quality to speed up diagnosis and treatment
Consumption	Precise promotion behavior analysis	Promote customer buying enthusiasm and comply with customers' buying habits
Energy	Centralized analysis of sensor array data in exploration and drilling	Reduce accident risk and optimize the exploration process

**Table 2:** The strategic combination between core enterprises and upstream SMEs.

		Middle and upstream enterprises	
		Action	No action
Core Enterprise	Guarantee	(Action, Guarantee)	(No Action, Guarantee)
	No guarantee	(Action, No guarantee)	(No Action, No guarantee)

## Data Availability

The data that support the findings of this study are available from the corresponding author upon reasonable request.

## References

[1] Kouvelis P., Zhao W. (2018). Who should finance the supply chain impact of credit ratings on supply chain decisions. *Manufacturing & Service Operations Management*.

[2] Martin J., Hofmann E. (2017). Involving financial service providers in supply chain finance practices[J]. *Journal of Applied Accounting Research*.

The article "Sustainable Trend of Big Data in Enterprise Supply Chain Under the Artificial Intelligence Green Financial System" was retracted in 2023. Reasons: unreliable results or conclusions; concerns about the data; concerns about the peer review; concerns about the citations.

[3] Thurner T. (2018). Supply chain finance and blockchain technology – the case of reverse securitisation. *Foresight*.

[4] Song H., Qiang L. U., Business S. O. (2017). The innovation of supply chain finance pattern based on virtual clusters:A case study of SJET[J]. *China Industrial Economics*.

[5] Chen B., Xu K. (2021). Credit risk assessment of e-commerce supply chain finance of SMEs based on dynamic reward and punishment perspective[J]. *Discrete Dynamics in Nature and Society*.

[6] Yan H. (2021). New model of food supply chain finance based on the Internet of things and blockchain[J]. *Mobile Information Systems*.

[7] Hassabis D., Kumaran D., Summerfield C., Botvinick M. (2017). Neuroscience-inspired artificial intelligence. *Neuron*.

[8] Miller T. (2017). Explanation in artificial intelligence: insights from the social sciences[J]. *Artificial Intelligence*.

[9] Institute M. (2017). Artificial intelligence:the next digital frontier[J]. *Information Security and Communications Privacy*.

[10] Krittanawong C., Zhang H. J., Wang Z., Aydar M., Kitai T. (2017). The present and future: artificial intelligence in precision cardiovascular medicine[J]. *Journal of the American College of Cardiology*.

[11] Li R., Zhao Z., Zhou X. (2017). Intelligent 5G: when cellular networks meet artificial intelligence. *IEEE Wireless Communications*.

[12] Varian H. (2018). Artificial intelligence, Economics, and industrial organization[J]. *Hal Varian*.

[13] Yeh J.-Y., Chen C.-H. (2020). A machine learning approach to predict the success of crowdfunding fintech project. *Journal of Enterprise Information Management*.

[14] Cai H. J., Guo Z. (2019). New framework of supply chain finance: blockchain& big data[J]. *Theoretical Investigation*.

[15] Wamba S. F., Angappa G. (2018). Big data analytics in logistics and supply chain management[J]. *International Journal of Logs Management*.

[16] Wu K. J., Liao C. J., Tseng M. L., Lim M. K., Hu J., Tan K. (2017). Toward sustainability: using big data to explore the decisive attributes of supply chain risks and uncertainties. *Journal of Cleaner Production*.

[17] Li L., Zhang J. (2021). Research and analysis of an enterprise E-commerce marketing system under the big data environment. *Journal of Organizational and End User Computing*.

[18] Venkatesh M., Delgado C., Patel P. (2017). Mitigating supply chain risk for sustainability using big data knowledge: evidence from the manufacturing. *Supply Chain*.

[19] Bag S. (2017). Big data and predictive analysis is key to superior supply chain performance: a South African experience[J]. *International Journal of Information Systems and Supply Chain Management*.

The article "Sustainable Trend of Big Data in Enterprise Supply Chain Under the Artificial Intelligence Green Financial System" was retracted in 2023. Reasons: unreliable results or conclusions; concerns about the data; concerns about the peer review; concerns about the citations.

[20] Sun Y., Li Li., Tian J. (2021). Research on the application of big data in regional industrial supply chain[J]. *Journal of Physics: Conference Series*.

[21] Niu B., Zou Z. (2017). Better demand signal, better decisions evaluation of big data in a licensed remanufacturing supply chain with environmental risk considerations. *Risk Analysis*.

[22] Tiwari S., Wee H. M., Daryanto Y. (2018). Big data analytics in supply chain management between 2010 and 2016: i. *Computers & Industrial Engineering*.

[23] Zaied A. N. H., Mohmed S. (2020). ERP implementation road Map for small and medium size enterprises (SMEs). *Journal of Intelligent Systems and Internet of Things*.

